# Comparison of the Accuracy of 3D Images Obtained fromDifferent Types of Scanners: A Systematic Review

**DOI:** 10.1155/2020/8854204

**Published:** 2020-12-14

**Authors:** Dorota Kustrzycka, Tim Marschang, Marcin Mikulewicz, Wojciech Grzebieluch

**Affiliations:** ^1^Division of Facial Abnormalities, Department of Maxillofacial Orthopedics and Orthodontics, Wroclaw Medical University, Wroclaw, Poland; ^2^Faculty of Dentistry, Wroclaw Medical University, Wroclaw, Poland; ^3^Department of Conservative Dentistry and Pedodontics, Wroclaw Medical University, Wroclaw, Poland

## Abstract

**Introduction:**

The purpose of this systematic review was to compare the accuracy of the three-dimensional images among different scanners, scanning techniques, and substrates. *Materials and methods*. Electronic databases (PubMed and Elsevier) were searched until March 2020. The systematic search was performed to identify the most precise method of obtaining a 3D image of the dentition.

**Results:**

Thirteen articles out of 221, considering the accuracy of 3D images, were selected. The main factors that are considered to have an influence on the precision are substrate type in the oral cavity, experience of the scanner's operator, direct vs. indirect scanning, and the reproducibility of the procedure.

**Conclusion:**

Substrate type does have an impact on the overall accuracy of intraoral scans where dentin has the most and enamel the least accurately recorded dental structure. Experience of the operator has an influence on the accuracy, where more experienced operators and smaller scan sizes are made for more accurate scans. A conventional impression technique in a full-arch image provided the lowest deviation. The reproducibility of direct scanning was comparable to indirect scanning although a slight difference was noticeable (0.02 mm).

## 1. Introduction

Nowadays, 5 to 10% of dentists use the possibility to get a digital dental impression of the dentition with the use of intraoral scanners, and the percentage rises every year [1]. In the last decade, digitalization has gained increasing importance in the everyday dental practice [2]. Conventional impressions are still very common. However, it is well known that digital models offer more advantages, for example, better precision while measuring the size of teeth, calculating the orthodontic indices, and collecting all data needed for the diagnosis [3]. Due to the possibilities which digitally collected data provides, additional perspectives arise, which, compared to conventional methods, would be complicated or sometimes not even be possible [4]. Even though we are in the digital era of dentistry, a lot of clinicians doubt whether intraoral scan can fully replace an impression. A group of researchers from Switzerland concluded that the digital technique yielded higher local deviations while scanning the complete-arch cast [5]. A Korean group of prosthodontists claim that the accuracy of an intraoral scanner is greater than a conventional method. However, it decreases as the size of the scan increases [6]. A fundamental change and advantage for patients are digital impressions, especially for those with strong vomiting reflexes [7]. In orthodontics, proper diagnosis, treatment follow-up, and interdisciplinary consultations require often transport of plaster cast which causes potential damage. Additionally, the need of storage stone models, 10 years after finishing treatment, demands from the practitioners a lot of physical space in their dental offices [7]. Digital casts include more efficient storage and retrieval, easier transferability, superior durability, increased diagnostic versatility, and decreased processing time [8]. On the contrary, the advantages of conventional materials are that they are accurate, less expensive, and well-accepted [9, 10].

Therefore, the question is what kind of scanner and method of scanning should be used in digital orthodontics to get the best results?

## 2. Materials and Methods

This systematic review was conducted following the Preferred Reporting Items for Systematic Reviews and Meta-Analyses (PRISMA) statement. The review was registered in PubMed and Elsevier databases. The literature search was independently conducted by two researchers (D.K., T. M) in March 2020, utilizing articles in English based on original studies. No time filter was used. The detailed search terms and strategy are presented in Table 1. The electronic search was complemented by a manual search of bibliographies from full-text articles and abstracts. Inclusion criteria were original articles in English, and exclusion criteria were systematic reviews, case reports, letters, and articles written in a different language than English.

### 2.1. PICOS Question

On the basis of Participants, Interventions, Comparisons, Outcomes, and Study (PICOS) design, the focus questions that guided this systematic review were which scanner is the most precise? What influences the precision of a digital image obtained from the scanning procedure? Does in vivo scanning provide better results than ex vivo scanning?

## 3. Results

Thirteen articles out of 221 considering the accuracy of 3D images were selected using inclusion criteria (Table 2). After reading all articles, only 13 of them were included in the study. Of the considered factors, the main ones that might have an influence on the precision are substrate type in the oral cavity, experience of the scanner's operator, direct vs. indirect scanning, and the reproducibility of the procedure.

## 4. Discussion

A study group from Korea [13] compared two 3D images collected from in vivo and ex vivo scans made of casts based on impressions using the TRIOS scanner (3 Shape). The researchers compared the images of patients with a full dentition, except third molars, and scanned patients twice, with an interval of two weeks. The results showed greater discrepancies in the posterior than in the anterior region of dental arch on the scanned images. The average surface difference between the first and second images in the in vivo scans was about 0.02 mm greater than that of the ex vivo equivalents. The accuracy of measurements while comparing alginate impressions to dental scans is mostly based on recordings of the posterior and anterior regions (intercanine and intermolar distances). A study from Korea (2016) showed that there is no difference between plaster models and intraoral scans, except for one measurement of the lower intermolar width. The average surface difference amounts to 0.10 mm. Therefore, the results indicate that intraoral scans are acceptable clinically and can be used instead of plaster models [14]. A similar study from Brazil (2017) was undertaken, where not only intercanine and intermolar distances but also tooth diameter and height, overjet, overbite, and the sagittal relationship were measured. The findings showed that the measuring method can affect the reproducibility of the measurements [11]. The type of scanned tissues was always a challenge in terms of reliability when obtaining anatomical structures. In Nijmegen, in 2018, researchers studied whether the accuracy of the shape, color, and curvature of palatal soft tissues can be obtained in the scanned image. The results support the hypothesis that an intraoral scan can record a 3D image of palatal soft tissues [16].

### 4.1. Substrate

Another questionable factor that could affect the scan is the type of substrate. The type of scanned tissue (substrate) does not impact the overall accuracy of intraoral scans, which is a hypothesis that was confirmed by researchers from South Carolina in 2019 [15]. However, researchers from the same region, but a year later, claimed that the type of substrate does affect the trueness and precision of a scan. They found that active triangulation scanners are more sensitive to substrate differences than their parallel confocal counterparts. Due to the advances in technology, some scanners scan certain substrates better, but, in general, the new generation of scanners has overcome the problems of the old, including a collective improvement in the imaging of all substrates [17].

Digital orthodontics provides more comfort to the patient, which was also found in a study conducted in London in 2019. Patients questioned after the procedure of scanning and having their impressions taken answered that scanning is more comfortable than the latter. However, it takes more time, as the clinician has to calculate the automated PAR (Peer Assessment Rating) scoring [12].

There was a study that compared 2 intraoral scanners: TRIOS 3, 3 Shape and CS 3600, Carestream. TRIOS 3 displayed slightly higher precision (approximately 10 *μ*m) compared to CS 3600, only after superimposition on the whole dental arch (*p* < 0.05). Both intraoral scanners showed good performance and comparable trueness (median: 0.0154 mm; *p* > 0.05). However, in individual cases and in various, not spatially defined areas, higher imprecision was evident. Thus, the intraoral scanners' appropriateness for highly demanding, spatially extended clinical applications remains questionable [18].

### 4.2. Experience of the Operator

Another aspect which is taken into account when comparing reproducibility and image trueness is the experience of the practitioner. Research from Seoul in 2018 showed that newer systems were less likely to be influenced by the length of clinical career as well as the region being scanned [19]. This theory was confirmed by studies from Seoul in 2017 and Brazil in 2020, though in the Brazilian study, the team of operators consisted of 3 professionals with different levels of experience in contrast to Seoul's research studies, which used assistants as operators [20].

### 4.3. Type of Scanner or Software

A study group from Giessen studied the transfer accuracy of four different scanners (Trios3Cart, Trios3Pod, Trios4Pod, and Primescan), which were equipped with the latest software versions. They compared obtained data to conventional impressions. What they received was that current IOSs equipped with the latest software versions demonstrated less deviation for short-span distances compared to the conventional impression technique. However, the results showed that, for long-span distances, the conventional impression technique provided the lowest deviation. “Overall, currently available IOS systems demonstrated improvement regarding transfer accuracy of full-arch scans in patients” [21]. Another research that compared different scanners was carried out in Freiburg in 2013. They compared an intraoral scanner (iTero) and an extraoral scanner (D250; 3Shape, Copenhagen, Denmark) and found that iTero was less accurate than scanning with the D250. This result suggests that the intraoral conditions (saliva, limited spacing) contribute to the inaccuracy of a scan. Intraoral scanners could be used for treatment planning and manufacturing of tooth-supported appliances [22].

A study from New York compared 4 intraoral optical scanners (True Definition, TRIOS, CEREC Omnicam, and Emerald Scanner) on an edentulous mandible model with 6 hexagonal scan bodies. There were neither statistical nor clinical differences among scanners [23].

## 5. Conclusions

Substrate type has an impact on the overall accuracy of intraoral scans, where dentin is the most and enamel is the least accurately recorded dental structure. The experience of the operator has an influence on the accuracy, where more experienced operators and smaller scan sizes make more accurate scans. A conventional impression technique in a full-arch recording provides the lowest deviation. The reproducibility of direct scanning is comparable to indirect scanning although a slight difference can be noticed (0.02 mm).

## Figures and Tables

**Table 1:** Search strategy.

1	Search (intraoral scanner AND orthodontics) AND precision) AND accuracy)

2	Search (intraoral scanner AND orthodontics)

3	Search (intraoral scanner) AND precision) AND accuracy)

**Table 2:** Selected articles.

Study	Title of the article	Description of the methodology	Search strategy
Dutton et al. [10]	The effect different substrates have on the trueness and precision of eight different intraoral scanners	A custom model, used as the reference standard, was fabricated with teeth composed of different dental materials; the reference standard scan was obtained using a three-dimensional (3D) optical scanner, the ATOS III; experimental scans were obtained using eight different IOS and operated by experienced clinicians using the manufacturer's recommended scanning strategy; a comprehensive metrology program, Geomagic Control X, was used to compare the reference standard scan with the experimental scans	intraoral scaner + orthodontics + precision + accuracy

Bocklet et al. [9]	Effect of scan substrates on accuracy of 7 intraoral digital impression systems using human maxilla model	Seven digital intraoral impression systems were used to scan a freshly harvested human maxilla; the maxilla contained several teeth restored with amalgam and composite, as well as unrestored teeth characterized by enamel; also, three teeth were prepared for full-coverage restorations to expose natural dentin; an industrial-grade metrology software program allowed 3D overlay and dimensional computation compared deviations of the complete arch and its substrates on the test model from the reference model	intraoral scanner + orthodontics + precision + accuracy AND intraoral scanner + orthodontics

Lim et al. [11]	Comparison of digital intraoral scanner reproducibility and image trueness considering repetitive experience	Twenty dental hygienists scanned 10 times his/her one assigned patient with Trios and iTero scanners, the superimposition of each patient was compared with, and Precision was calculated as the mean deviation among all superimposition combinations from the 10 scanned data sets of each learner [*n* = 10C2 = 45]; trueness was evaluated by superimposing the 10 consecutive intraoral scan data onto the impression scan data from each patient's rubber impression body (*n* = 10)	intraoral scanner + orthodontics + precision + accuracy AND intraoral scanner + orthodontics

Flügge et al. [12]	Precision of intraoral digital dental impressions with iTero and extraoral digitization with the iTero and a model scanner	One patient was scanned 10 times with iTero scanner and had impression taken (intraoral scan, group 1); next, his stone cast was scanned 10 times with iTero, group 2, and 10 times with extraoral model scanner, group 3	intraoral scanner + orthodontics + precision + accuracy
Luqmani et al. [13]	A comparison of conventional vs. automated digital Peer Assessment Rating scoring using the Carestream 3600 scanner and CS Model + software system: a randomized controlled trial	The sample consisted of 67 patients; mean age 15.03 (range 11–37) years; sixty-seven patients underwent alginate impression-taking and intraoral scanning (CS 3600; Carestream Dental, Stuttgart, Germany) at a single appointment in a randomized order; for each patient, a weighted PAR score was calculated manually by a calibrated examiner using study models and a PAR ruler (conventional group) and automatically using Carestream Dental CS Model + software and data from scanned study models (indirect digital group) or intraoral scans (direct digital group); all procedures were timed, and each patient completed a binary questionnaire relating to their experience	intraoral scanner + orthodontics

Winkler and Gkantidis [14]	Trueness and precision of intraoral scanners in the maxillary dental arch: an in vivo analysis	In 12 subjects, we evaluate the trueness and precision of two widely used intraoral scanners (TRIOS 3, 3Shape, and CS 3600, Carestream), using an industrial scanner (Artec Space Spider) as a reference; trueness of the intraoral scans was analyzed by measuring their distance from the reference scan, in the upper buccal front area; precision was tested through the distance of repeated scans regarding the whole dental arch, following superimpositions in the buccal front and in the whole dental arch area	intraoral scanner + orthodontics

Sun et al. [5]	Reproducibility of an intraoral scanner: a comparison between in vivo and ex vivo scans	Twenty adults with no missing teeth except for third molars were included in the study; alginate impressions were taken, and plaster models were made from the impressions; each subject underwent full-arch intraoral scanning twice with a TRIOS scanner (3Shape, Copenhagen, Denmark) at an interval of 2 weeks, and the plaster models were scanned at the same interval with the same scanner; the first images of each scan were superimposed on the second scanned images using surface-based registration; in each case, the differences between the 2 scanned images were evaluated with color mapping; the reproducibility between the in vivo and ex vivo scans was compared using independent *t* tests and Bland–Altman analysis	intraoral scanner + orthodontics
Deferm et al. [8]	Validation of 3D documentation of palatal soft tissue shape, color, and irregularity with intraoral scanning	Intraoral scans of ten participants' upper dentition and palate were acquired with the TRIOS® 3D intraoral scanner by two observers; conventional impressions were taken and digitized as a gold standard; the resulting surface models were aligned using an Iterative Closest Point approach; the absolute distance measurements between the intraoral models and the digitized impression were used to quantify the trueness and precision of intraoral scanning; the mean color of the palatal soft tissue was extracted in HSV (hue, saturation, and value) format to establish the color precision; finally, the mean curvature of the surface models was calculated and used for surface irregularity	intraoral scanner + orthodontics

Camardella et al. [7]	Accuracy and reproducibility of measurements on plaster models and digital models created using an intraoral scanner	This study included impressions of 28 volunteers; alginate impressions were used to make plaster models, and each volunteers' dentition was scanned with a TRIOS Color intraoral scanner; two examiners performed measurements on the plaster models using a digital caliper and measured the digital models using Ortho Analyzer software; the examiners measured 52 distances, including tooth diameter and height, overjet, overbite, intercanine, and intermolar distances, and the sagittal relationship; the paired *t* test was used to assess intraexaminer performance and measurement accuracy of the two examiners for both plaster and digital models; the level of clinically relevant differences between the measurements according to the threshold used was evaluated, and a formula was applied to calculate the chance of finding clinically relevant errors on measurements on plaster and digital models	intraoral scaner + orthodontics
Zhang et al. [6]	Validity of Intraoral Scans Compared with Plaster Models: An In Vivo Comparison of Dental Measurements and 3D Surface Analysis	Two types of dental models (intraoral scan and plaster model) of 20 subjects were included in this study; the subjects had impressions taken of their teeth and made as a plaster model; in addition, their mouths were scanned with the intraoral scanner, and the scans were converted into digital models; eight transverse and 16 anteroposterior measurements, 24 tooth heights, and widths were recorded on the plaster models with a digital caliper and on the intraoral scan with 3D reverse engineering software	intraoral scanner + orthodontics

Schmidt et al. [15]	Accuracy of Digital and Conventional Full-Arch Impressions in Patients: An Update	Trueness/precision of four intraoral scanners was assessed in five patients versus conventional impressions	intraoral scanner + precision + accuracy

Resende et al. [16]	Influence of operator experience, scanner type, and scan size on 3D scans	Trueness and precision of scans performed by 3 professionals with different levels of experience by using 2 IOSs were evaluated	intraoral scanner + precision + accuracy

Sami et al. [17]	An in vitro 3D evaluation of the accuracy of 4 intraoral optical scanners on a 6-implant model	Four IOSs scanned a 6-implant model each five times, and the trueness and precision were assessed afterwards	intraoral scanner + precision + accuracy

## Data Availability

No data were used to support the findings of the study.
